RETRACTED

# Neurological Manifestations of Infectious Diseases: Insights From Recent Cases

**DOI:** 10.7759/cureus.51256

**Published:** 2023-12-28

**Authors:** Jyoti Kashyap, Olusegun A Olanrewaju, Kinza Mahar, Meena Israni, Reena Bai, Narendar Kumar, Komal Kumari, Sujeet Shadmani, Muhammad Arsalan Bashir, Mostafa Elharif, Giustino Varrassi, Satish Kumar, Mahima Khatri, Muhammad Ali Muzammil, Roshan Sharma, Farhan Ullah

**Affiliations:** 1 Medicine, Sri Balaji Action Medical Institute, Delhi, IND; 2 Pure and Applied Biology, Ladoke Akintola University of Technology, Ogbomoso, NGA; 3 General Medicine, Stavropol State Medical University, Stavropol, RUS; 4 Medicine, Bahria University Medical and Dental College, Karachi, PAK; 5 Medicine, Sir Syed College of Medical Sciences, Karachi, PAK; 6 Medicine, Liaquat University of Medical and Health Sciences, Jamshoro, PAK; 7 Internal Medicine, Burjeel Hospital, Abu Dhabi, ARE; 8 Medicine, NMC Royal Family Medical Centre, Abu Dhabi, ARE; 9 Medicine, Shaheed Mohtarma Benazir Bhutto Medical College, Karachi, PAK; 10 Medicine, Ziauddin University, Karachi, PAK; 11 Medicine, Menoufia University, Shibin El Kom, EGY; 12 Pain Medicine, Paolo Procacci Foundation, Rome, ITA; 13 Internal Medicine/Cardiology, Dow University of Health Sciences, Karachi, PAK; 14 Internal Medicine, Dow University of Health Sciences, Karachi, PAK; 15 Medicine, Sanjay Gandhi Memorial Hospital, Delhi, IND; 16 Internal Medicine, Khyber Teaching Hospital, Peshawar, PAK

**Keywords:** parasites, bacteria, virus, infectious, neurological

## Abstract

This narrative review examines the complex connection between infectious diseases and their neurological effects. It provides a detailed analysis of recent instances and insights derived from various pathogens. As we explore the realm of infectious agents, including viruses, bacteria, parasites, and fungi, a thorough and diverse analysis reveals the intricacies of neurological problems. The review begins by examining viral infections, specifically focusing on how viruses invade the neurological system and its subsequent effects. Significant instances from recent widespread disease outbreaks function as instructive benchmarks, highlighting the progressing comprehension of these ever-changing interconnections. The article examines the complex pathophysiology of neurological problems caused by bacterial infections. It presents current cases that illustrate the various ways these complications might manifest and the difficulties faced in their therapeutic management. Parasitic and fungal infections, which are typically overlooked, are being carefully examined to emphasize their distinct role in causing neurological complications. The mentioned cases highlight the importance of being thoroughly aware of these less-explored areas ranging from protozoan parasites to opportunistic fungal infections. In addition to the immediate effects caused by infectious agents, the review investigates autoimmune responses activated by infections. It provides a detailed examination of specific instances that shed light on the complex relationship between viral triggers and future neurological problems. This text elaborates on the intricacy of autoimmune-related neurological issues, highlighting the necessity for a comprehensive approach to diagnosing and treating them. The narrative next redirects its attention to the diagnostic difficulties that arise when interpreting the neurological symptoms of viral disorders. This article provides a thorough examination of existing diagnostic tools, along with an investigation into new technologies that have the potential to improve our capacity to identify and comprehend complex presentations. This debate connects to the following examination of treatment methods, where current cases that showcase successful interventions are carefully examined to extract valuable insights into good clinical management. The discussion focuses on the public health implications of preventive efforts against infectious infections, including their neurological consequences. The story emphasizes the link between infectious diseases and overall societal health, advocating for a proactive strategy to reduce the impact of neurological complications. The abstract concludes by providing a prospective viewpoint, highlighting areas of research that still need to be addressed, and suggesting potential future avenues. This narrative review seeks to provide a comprehensive resource for physicians, researchers, and public health professionals dealing with the complex field of neurological manifestations in infectious diseases. It combines recent examples, synthesizes current information, and offers a holistic perspective.

RETRACTED

## Introduction and background

The connection between viral infections and neurological symptoms has recently become an essential area of study in medical research. The complicated interaction between viruses and the central nervous system has revealed numerous intricacies beyond the usual limits of managing infectious diseases [1]. This narrative review explores the complex nature of neurological manifestations of infectious diseases (NMID) by analyzing the knowledge gained from recent cases. Both physicians and researchers must have a thorough grasp of this relationship. It not only helps reveal the underlying pathophysiological mechanisms of these difficulties but also has significant consequences for creating specific treatment strategies [2]. The correlation between infectious diseases and neurological symptoms is a topic of growing importance in the medical field. Contagious diseases have historically been linked to systemic symptoms such as fever, fatigue, and dysfunction in specific organs [3]. Nevertheless, acknowledging the nervous system as a principal target for many pathogens has expanded our comprehension of disease pathophysiology. Recent instances have highlighted the capacity of infectious agents to cross the blood-brain barrier or enter the central nervous system through several pathways, resulting in a range of neurological problems varying from slight cognitive decline to severe brain disorders [4]. Given the ongoing changes in global infectious illnesses, understanding the complex relationship between hosts and pathogens is crucial for developing practical therapeutic approaches.

Understanding the neurological consequences of viral diseases is important beyond mere academic interest. The clinical significance is essential, as neurological symptoms can significantly add to the illness and death rates associated with infectious illnesses [5]. Moreover, the intricate and varied characteristics of these problems present difficulties in diagnosis, necessitating a heightened level of knowledge among healthcare professionals. The failure to promptly identify and tackle NMID can result in enduring repercussions such as permanent neurological harm and persistent impairment. In the face of new and dangerous infectious diseases, it is crucial to have a detailed understanding of their neurological consequences [6]. This knowledge is essential for developing effective public health strategies and clinical recommendations. The narrative review aims to fill the current knowledge vacuum and provide the medical community with valuable insights that have significant consequences for patient care and global health outcomes. This narrative review aims to consolidate and examine the large amount of material obtained from recent cases, providing a thorough summary of the changing landscape of NMID. The study seeks to understand the pathophysiological basis of neurological problems by examining the complex interactions between infectious agents and the nervous system [7]. Furthermore, it aims to recognize similarities and differences among various contagious agents, providing insights into possible treatment targets and prevention measures. The amalgamation of several case studies offers a nuanced viewpoint beyond specific factors related to individual pathogens, presenting a comprehensive framework for comprehending the broader consequences of NMID [8].

RETRACTED

This narrative review aims to contribute substantially to the existing knowledge about the neurological symptoms of viral illnesses. The study examines the complexities of this delicate interaction, improving our understanding of how diseases develop and highlighting the crucial need for a multidisciplinary approach in handling these complex clinical situations. As the world deals with the ever-changing nature of infectious diseases, the findings from this analysis can provide valuable information for evidence-based therapies. This can help advance medical understanding and enhance patient outcomes.

## Review

Methodology

The methodology utilized in the inquiry, "Neurological Manifestations of Infectious Diseases: Insights From Recent Cases," is carefully crafted to guarantee an intense and all-encompassing examination. The selection criteria for current cases are of the utmost importance in establishing the basis of this research. "Recent cases" refers to those recorded in the past five years. Given the constantly changing nature of infectious diseases, this timeframe was specifically chosen to ensure that the data collected is up-to-date and relevant. This temporal criterion aims to integrate the most recent clinical, diagnostic, and therapeutic breakthroughs to gain a detailed understanding of the neurological symptoms related to viral disorders. The screening method also required that selected instances be published in peer-reviewed journals or credible medical databases. The strict standard guarantees the dependability and trustworthiness of the documented cases since scholarly material is subjected to a comprehensive assessment conducted by specialists in the respective domain. The research attempts to uphold a rigorous standard of evidence and make a meaningful contribution to the current knowledge on the issue by exclusively focusing on reliable sources. Another crucial factor in selecting cases is the verification of the diagnosis. Chosen points should exhibit a distinct and thoroughly documented diagnosis, encompassing the infectious disease and the related neurological symptoms. Adhering to this criterion is crucial in maintaining the reported information's precision and reliability, reducing the possibility of misinterpretation or the inclusion of instances that need a more robust diagnostic basis.

Furthermore, the study incorporates instances encompassing different infectious agents to provide a thorough understanding of the vast array of viral disorders and their neurological consequences. The chosen cases encompass a range of bacteria, viruses, fungi, and parasites, representing the diverse assortment of pathogens that can impact the central nervous system (CNS). This criterion improves the study's ability to obtain comprehensive insights into the similarities and differences in neurological symptoms among various viral illnesses. The study includes a wide range of infectious agents and examines variations in demographics. Including cases from various age groups and demographics allows for considering potential differences in neurological symptoms based on characteristics such as age, gender, and geographical location. This methodology guarantees that the results are representative and appropriate to various individuals, recognizing that neurological symptoms may differ among multiple demographic cohorts. The search approach for locating relevant material follows the recommendations of the scale for the quality assessment of narrative review articles (SANRA). The systematic method ensures transparency and rigor in conducting a literature review. The initial stage is identifying keywords associated with infectious diseases and neurological symptoms to provide a thorough and focused search. Working together with medical librarians improves the accuracy of the search strategy, optimizing the choice of relevant keywords, and maximizing the retrieval of related literature.

RETRACTED

Selecting the appropriate databases is a critical component of the search strategy. PubMed, MEDLINE, Embase, and other pertinent medical databases were thoroughly queried to discover papers that fulfilled the study's requirements. The deliberate incorporation of multiple databases is intended to mitigate the possibility of disregarding pertinent material and to ensure a comprehensive examination of the current knowledge base. The search strategy includes grey literature such as conference proceedings and reports. Undertaking this step is crucial to encompass a broader spectrum of recent instances that might not be documented in conventional peer-reviewed publications. The study seeks to incorporate grey literature to access a more comprehensive dataset, acknowledging that valuable insights can be obtained from sources other than traditional academic publications. Boolean operators are employed to further narrow search queries, increasing the results' specificity. The deliberate utilization of AND, OR, and NOT operators guarantees that the search results closely correspond to the study's goals, hence aiding the detection of pertinent material while avoiding extraneous or duplicative data.

Hand-searching of journals is a supplementary measure in the search strategy entailing a manual examination of pertinent journals and their archives. This methodical approach enhances the electronic search by acting as a system of checks and balances to identify cases that may not be included in electronic databases. The manual examination is performed with meticulous attention guaranteeing that no potential source of information is disregarded. The criteria used to determine which cases are included or excluded are essential elements of the methodological framework. The purpose of inclusion criteria is to uphold the rigor and concentration of the investigation, prioritizing characteristics that enhance the pertinence and dependability of the chosen examples. For a case to be considered, it must meet the following requirements: it must have been published in the past five years, it must include a detailed and thorough diagnosis of both the infectious disease and the related neurological symptoms, and it must come from reliable sources such as peer-reviewed journals or recognized medical databases. In contrast, exclusion criteria are implemented to eliminate cases that do not correspond to the study's objectives or do not fulfill the set requirements. Excluded are issues that do not have a definitive diagnosis of the infectious disease or neurological manifestation, guaranteeing that only cases with thoroughly documented and indisputable diagnoses are considered. Likewise, instances without adequate clinical information for significant analysis are removed to uphold the study's findings' integrity.

RETRACTED

In addition, the study does not include papers not published in peer-reviewed journals or renowned medical databases. This criterion strengthens the dedication to obtaining reliable and credible evidence, prioritizing sources that have undergone thorough and rigorous evaluation by experts in the field. Instances involving neurological manifestations not associated with infectious diseases are also disregarded as the research specifically concentrates on the connection between infectious diseases and neurological consequences. In order to mitigate potential biases and provide a targeted investigation, the study employs exclusion criteria for cases that have incomplete or confusing information. This prudent methodology guarantees that the chosen instances offer a significant contribution to the study's goals while also preventing the inclusion of cases that could introduce confounding variables or uncertainties. The methods used to investigate the neurological symptoms of viral illnesses demonstrate a comprehensive and rigorous approach. The study's robustness and validity are enhanced by the careful selection of cases, adherence to the SANRA recommendations for the search approach, and the application of specific inclusion/exclusion criteria. The research seeks to offer detailed insights into the latest neurological symptoms linked to infectious diseases by following these methodological principles. This will significantly contribute to the current understanding of the field.

RETRACTED

General overview of infectious diseases and the nervous system

Infectious diseases encompass illnesses caused by harmful microorganisms including bacteria, viruses, fungi, and parasites [1]. These diseases can have significant effects on the brain system. The intricate interaction between infectious agents and the nervous system is a crucial field of research considering the diverse neurological symptoms that can arise from infections [2]. This section offers a broad introduction to infectious diseases and their possible effects on the nervous system. It explores the various ways infections can occur and the typical methods via which pathogens can infiltrate this complex and essential physiological system. Infectious diseases provide a worldwide health threat, impacting populations regardless of geographical or demographic distinctions. They originate from the infiltration of the body by pathogenic microbes, resulting in disruptions to regular physiological processes [3]. The nervous system, which consists of the CNS and peripheral nervous system (PNS), is susceptible to the effects of infectious attacks. Infections can lead to a range of neurological symptoms, varying from little cognitive decline to critical, life-threatening illnesses [4]. The pathways by which pathogenic pathogens enter the nervous system are varied, reflecting the intricate anatomical and physiological defenses that safeguard this crucial system. Hematogenous dissemination is the most frequent pathway, wherein infections enter the bloodstream and cross the blood-brain barrier (BBB) to access the CNS [5]. The BBB, composed of endothelial cells lining cerebral blood arteries, often limits the entry of infections and giant chemicals into the brain. Nevertheless, specific pathogens can penetrate this protective barrier, resulting in illnesses within the CNS [6].

Furthermore, infections can infiltrate the nervous system by entering the body directly by retrograde axonal transport. This process entails the infiltration of pathogens through nerve endings located in the periphery, followed by their transportation along nerve fibers toward the CNS [7]. Neurotropic viruses, including herpesviruses, frequently use this invasion method to develop hidden infections in the sensory ganglia. They can later reactivate, leading to neurological symptoms. An infrequent yet extremely significant method of infection occurs through the cerebrospinal fluid (CSF). The CSF flows across the subarachnoid space as a conduit for transmitting diseases within the CNS [8]. Meningitis, a condition that primarily affects the CSF, is characterized by inflammation of the meninges surrounding the brain and spinal cord. It can lead to neurological consequences. Interestingly, certain infections display tropism towards particular parts of the nervous system [9]. For example, the olfactory nerve is a direct pathway for some viruses to enter the brain, resulting in encephalitis. This behavior is observed in infections such as influenza, where the virus enters through the nasal mucosa and then infiltrates the olfactory nerve, resulting in neurological consequences [10].

RETRACTED

The means through which infections overcome the substantial barriers of the nervous system are complex and frequently employ sophisticated tactics to avoid detection by the immune system [10]. Viruses, renowned for their ability to undergo fast mutations, can acquire mechanisms to elude immune recognition and endure within cerebral tissues. In contrast, bacteria can generate poisons or utilize adhesion molecules to enhance their attachment to and invasion of host cells [11]. Within viral infections, specific viruses demonstrate neurotropism, which signifies an innate capacity to infect brain cells. Herpesviruses, such as herpes simplex virus (HSV) and varicella-zoster virus (VZV), are noteworthy instances of neurotropic viruses that can form latent infections in brain tissues [12]. These viruses can result in various neurological illnesses, varying from minor peripheral neuropathies to severe encephalitis. Meningitis, an inflammation of the meninges surrounding the brain and spinal cord, can be caused by bacterial infections such as *Neisseria meningitidis* or *Streptococcus pneumoniae* [13]. Bacterial entry into the CNS is aided by multiple mechanisms, such as the secretion of enzymes that break down host tissues. This enables the pathogens to overcome anatomical barriers and access the CNS [13].

Fungal infections, however less prevalent, can also affect the neurological system, especially those with weakened immune systems. *Cryptococcus neoformans*, for example, is a fungus that can cause meningitis in those with weakened immune systems [14]. The capacity of fungi to spread throughout the CNS underscores the wide array of infectious pathogens that can impact neurological function. Parasitic illnesses, while commonly linked to systemic symptoms, can also result in neurological complications [15]. *Toxoplasma gondii*, a type of single-celled parasite, can create tiny protective sacs called cysts in the neural tissues of the body. This can result in the development of neurological symptoms in people who have weaker immune systems [16]. Likewise, the single-celled organism *Trypanosoma cruzi*, which causes Chagas disease, can infiltrate the CNS, leading to neurological problems. Infectious diseases present a substantial risk to the nervous system, capable of inducing a wide range of neurological symptoms [17]. The varied infection pathways demonstrate the delicate interaction between pathogens and the complex anatomical and physiological barriers that protect the nervous system. Gaining insight into the paths via which infectious agents infiltrate the neural system is essential for developing precise treatment approaches and improving our ability to reduce the neurological effects of infections [18]. This comprehensive overview emphasizes the significance of ongoing research in elucidating the intricacies of viral disorders and their influence on neurological well-being.

RETRACTED

Neurological manifestations in infectious diseases

Neurological symptoms in viral diseases are complex and challenging to study and treat in medicine. This section classifies and examines distinct neurological symptoms, such as meningitis, encephalitis, neuropathies, and others, about various infectious diseases [19]. Moreover, the presentation of recent instances exemplifies the wide range of neurological problems linked to infectious agents, offering valuable insights into the intricacies of these interactions.

Meningitis

Meningitis is a notable neurological symptom in infectious disorders, where the meninges protecting the brain and spinal cord become inflamed. Bacterial meningitis, frequently triggered by organisms such as *N. meningitidis*, *S. pneumoniae*, and *Haemophilus influenzae*, has the potential to result in significant neurological consequences [20]. These bacteria commonly enter the CNS by traveling through the bloodstream, breaking through the BBB, and causing inflammation of the meninges. Recent cases underscore the sudden appearance of symptoms, such as intense headaches, high body temperature, and rigidity in the neck, highlighting the importance of promptly diagnosing and intervening [21]. Enteroviruses, herpesviruses, and arboviruses are recognized as the main causative agents of viral meningitis in the setting of viral infections. Enteroviruses, such as coxsackievirus and echovirus, frequently cause aseptic meningitis, characterized by a less severe progression than bacterial meningitis [22]. Recent examples highlight the significance of distinguishing between viral and bacterial causes as the treatment and outlook vary dramatically.

Encephalitis

Encephalitis is a medical condition characterized by inflammation of the brain. Encephalitis, characterized by inflammation of the brain tissue, manifests as a more severe type of neurological complication in infectious disorders. The HSV, namely HSV-1, is a primary factor in the development of viral encephalitis [21]. Recent examples have shown the swift advancement of symptoms, such as changes in mental state, seizures, and specific neurological impairments. Prompt diagnosis is crucial in controlling HSV encephalitis, emphasizing the significance of early antiviral treatment. Arboviruses, including West Nile virus and Japanese encephalitis virus, are significant contributors to viral encephalitis on a global scale [22]. Recent examples have demonstrated the wide range of neurological problems that can occur due to arboviral infections. These complications can vary from mild encephalitis to more severe results, such as paralysis and cognitive impairment [23]. The global distribution of arboviruses underscores the importance of adopting a worldwide approach to comprehending and controlling these contagious illnesses.

RETRACTED

Neuropathies

Neuropathies, which result in harm to peripheral nerves, are widespread in numerous infectious disorders. Guillain-Barré syndrome (GBS), a prime illustration of infectious neuropathy, is frequently instigated by infections such as *Campylobacter jejuni*, *Mycoplasma pneumoniae*, and Zika virus [24]. Recent cases have brought attention to progressive muscle weakness, a defining feature of GBS, emphasizing the importance of providing breathing assistance and initiating immunomodulatory treatment early. Human immunodeficiency virus (HIV)-related neuropathies, such as distal sensory polyneuropathy and HIV-related neuropathic pain, are essential consequences in patients with HIV infection [25]. Recent cases have clarified the persistent nature of these nerve disorders, which significantly damage the well-being of those affected. Antiretroviral therapy has shown effectiveness in preventing and treating HIV-related nerve disorders, highlighting the significance of comprehensive care in infectious diseases [26].

Cerebrovascular Complications

In addition, infectious infections can have a role in the development of cerebrovascular problems, such as stroke. Bacterial endocarditis, commonly triggered by *Streptococcus viridans *or *Staphylococcus aureus*, has the potential to result in embolic strokes [27]. Recent instances underscore the complex connection between infective endocarditis and neurological consequences, underscoring the importance of preventive actions in averting these complications. Malaria, an infection caused by parasitic Plasmodium species, is known for its ability to induce cerebral malaria, a severe form characterized by convulsions, coma, and localized neurological abnormalities [28]. The importance of promptly identifying and treating malaria to prevent permanent brain harm is underscored by recent occurrences. The significance of infectious infections in causing stroke highlights the necessity of employing a multidisciplinary strategy when treating patients with neurological problems [28].

RETRACTED

Neurological Consequences of COVID-19

The current COVID-19 pandemic, caused by the SARS-CoV-2 virus, has drawn attention to neurological symptoms. Recent cases have brought attention to the correlation between COVID-19 and neurological disorders, such as encephalopathy, acute disseminated encephalomyelitis (ADEM), and GBS [29]. The ability of SARS-CoV-2 to affect the nervous system raises worries regarding the long-term neurological consequences in persons who are recovering from COVID-19 [30].

Bacterial meningitis: A recent instance entailed a once-healthy young adult who exhibited a sudden and intense headache, sensitivity to light, and stiffness in the neck [31]. The CSF study revealed bacterial meningitis, and the timely delivery of suitable medicines resulted in a positive outcome. This case highlights the significance of promptly identifying and managing bacterial meningitis to avoid severe neurological complications [31].

HSV encephalitis: A case report describes an older adult who exhibited symptoms of disorientation, specific neurological impairments, and seizures. The study identified HSV-1 as the causal agent of CSF. Commencing antiviral medication promptly led to a steady amelioration of neurological symptoms [32]. This example emphasizes the need for timely diagnosis and focused antiviral therapy in managing HSV encephalitis.

Campylobacter infection-induced GBS: A person gradually loses strength and sensation in their limbs after contracting a gastrointestinal illness caused by *C. jejuni*. The diagnosis of GBS was established through electrophysiological testing [33]. Promptly administering immunomodulatory medication was crucial in substantially improving the patient's condition. This example demonstrates the correlation between viral triggers and the occurrence of neuropathies such as GBS [33].

COVID-19 has been linked to neurological complications. A recent case study described a patient who had COVID-19 and experienced sudden confusion, delirium, and indications of encephalopathy. Neuroimaging and analysis of CSF fluid excluded alternative explanations, indicating that SARS-CoV-2 is responsible for the observed neurological symptoms [34]. This example highlights the wide range of neurological problems linked to COVID-19. It emphasizes the importance of alertness in identifying these symptoms in clinical settings. Neurological symptoms in infectious disorders cover many consequences, including meningitis, encephalitis, and different neuropathies [35]. Recent instances offer valuable insights into how viral pathogens affect the neurological system, highlighting the significance of prompt diagnosis and focused therapies [35]. Continual research and a multidisciplinary approach are required to improve patient outcomes and deepen our understanding of the complicated interactions between viral illnesses and the nervous system [36].

RETRACTED

Pathophysiological mechanisms

The pathophysiological mechanisms that cause neurological problems in viral diseases are intricate and diverse. This section examines the complex interaction between infectious agents and the nervous system, providing insight into how infections penetrate protective barriers, trigger inflammation, and provoke immunological responses that result in neurological symptoms [36].

Disruption of the BBB

The BBB acts as a solid protective mechanism that controls the movement of chemicals between the bloodstream and the CNS. Several pathogens have developed tactics to penetrate the BBB, allowing them to enter the CNS and induce neurological symptoms [37]. *N. meningitidis* and *S. pneumoniae*, which are bacterial infections, can generate enzymes that break down tight junctions [37]. This action leads to the disruption of the integrity of the BBB. This break facilitates the entry of microorganisms into the brain, triggering inflammatory reactions that result in illnesses such as meningitis and encephalitis [37]. Neurotropism refers to the phenomenon where certain infections naturally prefer brain tissues. Herpesviruses, such as the HSV and VZV, are neurotropic viruses specifically targeting the nervous system. These viruses create dormant infections in the sensory ganglia and can reawaken, leading to neurological problems [38]. The processes for neurotropism entail the viruses' capacity to avoid immune detection and establish long-lasting infections in neurons. The delicate equilibrium between latency and reactivation plays a role in the recurring character of neurological symptoms caused by herpesviruses [38].

Retrograde Axonal Transport

Certain viruses utilize retrograde axonal transport to infiltrate the neurological system. The PNS is a pathway for pathogens to enter the CNS by traveling backward along nerve fibers. Neurotropic viruses, such as poliovirus and rabies virus, employ this technique [39]. For example, the rabies virus gains access to the CNS by utilizing retrograde axonal transport, which travels from the peripheral nerves to the spinal cord and brain. This mode of transportation enables the swift spread of the virus throughout the nervous system, resulting in severe neurological consequences [40].

RETRACTED

Inflammation in the CNS

Infections frequently provoke inflammatory reactions in the CNS, which play a role in developing neurological symptoms. Cytokines, chemokines, and immune cells coordinate these reactions. Bacterial infections, such as those causing meningitis, trigger a robust inflammatory response marked by the migration of immune cells into the CSF [41]. The presence of this inflammatory environment might lead to increased pressure inside the skull and contribute to symptoms related to the nervous system. Likewise, viral infections such as encephalitis caused by herpesviruses or arboviruses provoke inflammatory reactions that can harm tissues and impair neurological function [42].

Autoimmune Reactions

Infectious agents can initiate autoimmune reactions contributing to neurological problems. GBS is a prime example where molecular mimicry plays a vital role. After being infected with specific infections, such as *C. jejuni* and cytomegalovirus, the immune system produces antibodies that attack the infectious agent and parts of the neurons outside the brain and spinal cord [43]. The occurrence of cross-reactivity causes the destruction of myelin and damage to the axons, which leads to the distinctive paralysis that is observed in GBS and progresses from the lower to the upper body [44].

Toxins and Neurological Damage

Some diseases release toxins that directly harm neural tissues, worsening neurological symptoms. The bacterium *Clostridium tetani *is the causative agent of tetanus. It generates a toxin known as tetanus toxin, which disrupts the transmission of nerve signals, resulting in muscle stiffness and spasms [44]. Likewise, the botulinum toxin generated by *Clostridium botulinum* can induce paralysis by obstructing the release of acetylcholine at neuromuscular junctions. The presence of these poisons emphasizes the wide range of mechanisms by which infectious pathogens might interfere with regular brain function [45].

Vascular Problems and Stroke

Infectious infections play a role in the development of vascular problems, hence elevating the likelihood of experiencing a stroke. Bacterial endocarditis, defined by vegetation growth on heart valves, can cause emboli that block cerebral blood arteries [46]. The dissemination of septic emboli into the bloodstream during bacterial endocarditis presents a specific danger, which can potentially lead to ischemic strokes. This demonstrates the complex connection between viral processes, vascular impairment, and neurological consequences [47].

RETRACTED

Immunosuppression can lead to opportunistic infections in the nervous system, especially those that target the immune system. HIV attacks explicitly CD4+ T cells, resulting in immunosuppression. As a result of the decreased immune response, opportunistic infections, including toxoplasmosis and progressive multifocal leukoencephalopathy (PML), are able to flourish within the CNS [47]. The subsequent neurological consequences emphasize the susceptibility of the nervous system when the immune function is weakened. Severe infections, particularly those caused by highly pathogenic viruses, can trigger cytokine storms. These are characterized by an overactive immune response that results in the excessive release of pro-inflammatory cytokines [48]. Within neurological symptoms, cytokine storms play a role in promoting neuroinflammation. They can potentially result in disorders such as ADEM [49]. The latest instances linked to COVID-19 have highlighted the possible contribution of cytokine storms in worsening neurological problems. Specific pathogens have been linked to persistent inflammatory disorders that impact the neurological system [50]. Lyme disease, caused by the bacterium *Borrelia burgdorferi*, can potentially result in chronic neuroborreliosis, a condition marked by ongoing inflammation in neural tissues. The pathogen's capacity to elude the immune response and generate long-lasting infections highlights the difficulties in controlling and treating these neurological consequences [51].

The pathophysiological pathways that cause neurological symptoms in viral disorders are varied and complex. The infections' capacity to penetrate protective barriers, trigger inflammation, and influence immune responses adds to the intricacy of these interactions [52]. A comprehensive comprehension of these systems is essential for formulating precise therapies and therapeutic methods to alleviate the neurological repercussions of viral illnesses. Future research endeavors should persist in elucidating the complexities of these pathophysiological mechanisms, yielding vital understandings of the prevention and treatment of infectious disorders that impact the nervous system [53].

Diagnostic approaches

Diagnostic methods for recognizing neurological symptoms in viral disorders are crucial for prompt and precise intervention. This part provides an overview of the current diagnostic approaches, discusses the difficulties in identifying neurological problems, and examines the latest breakthroughs in diagnostic technologies. Gaining a thorough knowledge of these diagnostic methods is essential for improving patient outcomes and deepening our understanding of the complex connection between illnesses and the neurological system [54].

RETRACTED

Existing Diagnostic Techniques

Neurological manifestations are diagnosed with a thorough clinical assessment. Neurological symptoms, such as headache, altered mental status, seizures, and focal impairments, guide the diagnosis approach [22]. Various pathogens may display unique clinical manifestations, requiring a comprehensive evaluation of the patient's medical background and a complete physical examination. Neuroimaging studies are essential for detecting structural abnormalities in the nervous system [24]. Magnetic resonance imaging (MRI) is highly advantageous for visualizing the anatomy of the brain and spinal cord. Contrast-enhanced imaging facilitates the identification of regions displaying inflammation, ischemia, or mass lesions linked to infectious diseases [26]. Computed tomography scans can also be used, particularly in urgent conditions such as suspected bacterial meningitis.

CSF analysis: Performing a lumbar puncture to analyze the CSF is an essential diagnostic step for neurological infections. The process of CSF evaluation entails evaluating the number of cells, concentration of proteins, and glucose levels [26]. Furthermore, microbiological analysis, encompassing culture and polymerase chain reaction (PCR) assays, may accurately detect infectious agents such as bacteria and viruses. An increased number of white blood cells and elevated protein levels can suggest inflammation in the CNS [26]. Serological tests are used to detect and identify antibodies or antigens that are linked to particular infectious pathogens. For instance, serological assays can identify antibodies against neurotropic viruses such as HSV and arboviruses. These tests help identify recent or prior infections and can help confirm the cause of neurological symptoms [27].

Electroencephalography: Electroencephalography (EEG) is a method used to record the brain's electrical activity. EEG, or electroencephalography, is a technique used to assess the electrical activity in the brain. It is beneficial in identifying anomalies related to seizures and encephalopathies [28]. EEG results in infectious illnesses can indicate patterns suggestive of viral encephalitis or seizures. Continuous electroencephalogram monitoring is especially advantageous in severely sick patients who have experienced changes in their mental state [29].

Neurophysiological investigations: Electrophysiological investigations, such as nerve conduction tests and electromyography, are crucial in assessing peripheral neuropathies [30]. These examinations can detect deviations in nerve conduction velocity and muscle reflexes, assisting in identifying disorders like GBS [31].

RETRACTED

Difficulties in diagnosing neurological symptoms: Non-specific symptoms frequently accompany neurological manifestations in viral disorders, complicating the diagnosis process. Numerous factors might cause headaches, fever, and changes in mental state [33]. Thus, it is essential to take a thorough approach to distinguish infectious reasons from other possible factors.

Overlap of clinical presentations: The clinical manifestations of various infectious pathogens can coincide, creating difficulties in identifying the precise pathogen accountable for neurological symptoms [35]. Both bacterial and viral illnesses can cause meningitis, and it can be challenging to differentiate between them based purely on clinical signs.

Optimal timing of diagnostic testing: The precise timing of diagnostic testing is crucial since any delays can significantly impact patient outcomes. For example, lumbar puncture may not be recommended in specific clinical situations, and it is essential to get CSF samples promptly for precise microbiological examination [36]. Striking a balance between the necessity for timely diagnosis and individual patient factors is an ongoing difficulty.

Restricted specificity of serological testing: Serological assays, however valuable, may exhibit a lack of specificity, resulting in false-positive outcomes. The presence of antibodies from past infections or cross-reactivity can make it challenging to interpret serological findings [37]. This poses a hurdle in establishing a conclusive connection between infectious pathogens and neurological symptoms. There is a significant range of differences in the imaging results among patients with neurological symptoms [38]. The variability in imaging patterns can be attributed to the dynamic character of infectious processes and the wide range of pathogens involved. Accurate diagnosis relies on the crucial task of interpreting imaging findings within the patient's clinical presentation framework [39].

Progress in Diagnostic Techniques

Molecular diagnostics, namely nucleic acid amplification techniques such as PCR, have significantly transformed the process of identifying infectious pathogens. Real-time PCR methods offer prompt and empathetic identification of viral genetic material in CSF, enabling early detection of neurotropic viruses [39]. Next-generation sequencing (NGS) refers to advanced technologies that facilitate thoroughly examining microbial genetic material. This enables the detection and identification of various pathogens present in clinical samples. NGS can reveal rare or newly emerging infectious pathogens and improve our comprehension of the range of microorganisms responsible for neurological symptoms [40]. Neuroinflammation biomarkers have become increasingly important in identifying specific indicators of inflammation. Elevated levels of interleukin-6 (IL-6) or tumor necrosis factor-alpha (TNF-α) in CSF can indicate the presence of inflammation. Using these biomarkers improves the accuracy of detecting inflammatory conditions in the CNS [41].

RETRACTED

Advanced imaging modalities: Sophisticated neuroimaging techniques, such as functional MRI (fMRI) and positron emission tomography scans, provide valuable information about the practical and metabolic characteristics of the brain [42]. These tools enhance our understanding of how infectious agents affect neuronal function and help us assess the level of neurological damage. Artificial Intelligence (AI) is used in image analysis, particularly in medical imaging, to aid in interpreting neuroimaging research [43]. Machine learning algorithms can analyze imaging data to detect patterns linked to particular infectious diseases. This has the potential to speed up the diagnosis process and improve the accuracy of diagnostic results [44]. Point-of-care testing refers to the use of technologies that allow for quick and immediate diagnostic evaluations at the location where the patient is being treated. These devices are handy in settings when resources are limited [45]. These portable devices can rapidly yield outcomes for specific infectious pathogens, enabling prompt clinical decision-making.

Advancements in biosensors and wearable technology: Novel technologies like biosensors and wearable devices present prospects for uninterrupted monitoring of physiological data [46]. For viral disorders that affect the nervous system, these technologies can offer immediate information on alterations in neurological function, enabling prompt intervention and tailored patient care [45].

Integration of diagnostic methods: The proper diagnosis of neurological symptoms in viral disorders typically requires the combination of various diagnostic methods. The integration of clinical assessment, neuroimaging, CSF analysis, and molecular diagnostics improves the accuracy of diagnosis and offers a comprehensive comprehension of the infectious mechanisms at play [46].

Examinations of specific instances: The chance to incorporate molecular diagnostics arose when a patient with acute encephalitis was encountered. PCR testing conducted in real-time on CSF samples promptly detected the presence of HSV DNA, thus proving its causative role [47]. This case emphasizes integrating molecular techniques for prompt and focused interventions.

RETRACTED

Neuroimaging analysis enhanced by AI: An AI-assisted examination of MRI scans helped identify modest abnormalities that suggested a specific infectious cause in a case of meningitis with unusual neuroimaging findings [48]. Incorporating AI technology in the interpretation of neuroimaging has shown the ability to improve diagnostic accuracy in challenging instances. Biomarker profiling for inflammatory conditions was demonstrated to be helpful in a case involving a patient with unexplained neurological symptoms [49]. The presence of increased levels of IL-6 and TNF-α in the CSF indicated the presence of an underlying inflammatory condition. This case highlights the importance of biomarkers in understanding the underlying mechanisms of neurological symptoms and directing specific treatment approaches [50].

Obstacles in the Execution

Although there have been notable breakthroughs in diagnostic technologies, obstacles remain in their widespread adoption. Barriers to the adoption of these technologies into ordinary clinical practice include issues such as accessibility, cost, and standardization of assays [51]. It is crucial to tackle these issues to guarantee fair access to sophisticated diagnostic methods in various healthcare environments. Diagnosing neurological symptoms in infectious diseases is constantly changing due to technological developments and a better understanding of how viruses and the nervous system interact [52]. An essential aspect of achieving precise and prompt diagnosis is the incorporation of clinical, imaging, and laboratory results through a multidisciplinary approach. Continued research endeavors and advancements in diagnostic technology provide the potential to enhance our capacity to detect and treat neurological problems linked to infectious infections [53]. Healthcare workers can improve patient outcomes and contribute to a more extensive understanding of the complex interaction between conditions and the nervous system by tackling hurdles and embracing developments [54].

Treatment strategies

Managing neurological problems resulting from infectious infections requires a sophisticated and thorough treatment strategy. This part offers a comprehensive examination of the existing treatment choices, investigates recent progress in therapeutic methods, and examines the outlook and possible lasting consequences for individuals with neurological symptoms [12]. Antimicrobial therapy is necessary to treat bacterial infections that cause meningitis or encephalitis rapidly. Empirical antibiotics are administered based on the probable pathogens until specific causative agents are determined through CSF investigation [13]. Customizing the treatment based on the identified pathogen is essential for achieving the best possible results. *N.* *meningitidis*-induced bacterial meningitis is commonly managed using intravenous ceftriaxone or cefotaxime [14]. Antiviral drugs are necessary for treating viral infections targeting the neurological system, such as HSV encephalitis. Acyclovir is the preferred treatment for HSV encephalitis and should be started promptly for optimal effectiveness. Antiviral medication aims to diminish virus replication, ease symptoms, and prevent long-term neurological complications [15]. Immunomodulatory therapy is crucial in treating immune-mediated neurological disorders such as GBS. Intravenous immunoglobulin (IVIG) or plasmapheresis aims to regulate the immune response, expedite recuperation, and reduce long-term neurological impairments [16]. The selection between IVIG and plasmapheresis is contingent upon clinical factors and the accessibility of the treatments.

RETRACTED

Anti-inflammatory drugs treat inflammatory conditions in the CNS [17]. Corticosteroids, such as dexamethasone, are used in autoimmune encephalitis to reduce inflammation and regulate the immune response. Ensuring a delicate equilibrium between the anti-inflammatory properties and possible adverse reactions is vital in treating these disorders [18]. Supportive care plays a crucial role in the management of neurological problems. This includes interventions such as analgesia, fluid administration, and assistance with breathing in severely unwell patients. Supportive therapies in cases of autonomic dysfunction are implemented to uphold essential bodily functioning and avert potential repercussions [19]. Surgical treatments may be required to address neurological problems caused by some infectious illnesses. For instance, abscesses in the brain may necessitate surgical drainage. In contrast, elevated intracranial pressure resulting from infections may indicate the requirement for neurosurgical procedures [20].

Recent Progress in Therapeutic Methods

Targeted antiviral medicines aim to create specific medications with improved effectiveness and fewer adverse effects. Foscarnet, brincidofovir, and nucleotide analogs that have an enhanced ability to enter the CNS exhibit potential in treating viral infections that affect the neurological system [21]. These developments improve the efficacy and tolerability of antiviral therapies. Immunotherapies are constantly advancing as researchers continue to investigate new drugs and methods [22]. Researchers are currently studying monoclonal antibodies targeting specific immunological pathways to treat disorders involving autoimmune or immune-mediated neurological consequences. The advancement of more detailed and focused immunomodulatory drugs has the potential to enhance therapeutic results and minimize adverse side effects [24].

RETRACTED

Methods for Precision Medicine

Precision medicine in infectious illnesses enables personalized treatment approaches that consider the patient's unique pathogen profile, immune response, and genetic factors. Personalized methods of antimicrobial and immunomodulatory medicines aim to maximize therapeutic effectiveness while minimizing negative side effects [34]. Neuroprotective techniques are becoming increasingly important in the field of infectious disorders that affect the nervous system [35]. Researchers are investigating substances that can preserve the nervous system, such as antioxidants and anti-inflammatory agents, to reduce harm to neurons and enhance results. These techniques are designed to target the enduring effects of infectious illnesses on brain function [36].

Advancements in pharmaceutical administration: The goal of advancements in drug delivery systems is to improve the precise delivery of treatments to the CNS. Nanoparticle-mediated drug delivery systems and novel formulations enhance drug permeation through the BBB, augmenting the accumulation of therapeutic agents at the specific location of infection or inflammation [38].

Implementation of telemedicine: The incorporation of telemedicine has become highly pertinent, particularly in worldwide health issues. Telemedicine enables the remote monitoring, consultation, and follow-up care of patients experiencing neurological symptoms due to infectious infections [39]. This method improves the availability of specialized medical treatment, guaranteeing continuous assistance for patients, even in distant or under-resourced areas.

Prognosis and long-term effects

Prognosis of Neurological Manifestations

The outlook for patients with neurological symptoms in infectious diseases varies greatly depending on factors such as the particular pathogen, the extent of neurological involvement, the promptness of treatment, and other existing health conditions [40]. The prompt and suitable intervention greatly impacts the results. In instances of severe cases, especially those pertaining to illnesses such as bacterial meningitis or viral encephalitis, the mortality rate might be significant [41]. Nevertheless, recent progress in critical care, antibiotic treatments, and supportive measures has led to enhanced rates of survival. The type and intensity of the neurological damage determines functional recovery after neurological difficulties. GBS and certain viral encephalitides can see significant improvement with prompt immunomodulatory treatments [42]. However, viral encephalitides may lead to lasting neurological impairments. After contracting viral disorders that affect the nervous system, cognitive and behavioral sequelae may occur in certain people. Even after the acute symptoms have been resolved, individuals may still experience persistent memory impairment, mood issues, and changes in behavior [43]. Post-infectious cognitive impairment is now being studied and is of significant interest in both scientific and therapeutic settings.

RETRACTED

Chronic Neurological Problems

Some viral infections, especially those with long-lasting or hidden stages, might result in enduring neurological problems [44]. Instances of chronic neurological Lyme disease are characterized by the persistence of symptoms even after receiving antibiotic therapy. Additionally, HIV-associated neurocognitive diseases might present as long-lasting cognitive impairment [44]. Neurological manifestations significantly impact the entire quality of life for individuals. Their ability to restore functional independence, manage persistent symptoms, and cope with potential psychosocial obstacles play a crucial role in determining their quality of life [45]. Rehabilitation therapies, psychosocial support, and long-term care planning are essential for maximizing these persons' quality of life [45].

Rehabilitation and Supportive Care

Rehabilitation therapies, such as physical, occupational, and speech therapy, are crucial in assisting persons with remaining neurological impairments. These interventions aim to increase functional autonomy, boost mobility, and target specific difficulties associated with cognition and communication [47].

Continued Surveillance

Sustained observation is crucial for evaluating the advancement of neurological symptoms, detecting developing problems, and modifying treatment strategies as needed. Regular neurological exams, neuroimaging studies, and cognitive tests are essential to comprehensive long-term care [48].

Examples of Specific Situations

Efficient rehabilitation after GBS: A case study including a patient diagnosed with GBS underscored the significance of promptly administering immunomodulatory medication [48]. The timely beginning of IVIG therapy had a crucial role in facilitating a substantial improvement in the patient's condition, leading to a near-complete restoration of normal bodily function. This instance highlights the beneficial effect of prompt intervention on the prognosis [49].

Chronic cognitive dysfunction post-encephalitis: Following a viral encephalitis episode, the patient's acute symptoms subsided, but they nevertheless displayed enduring cognitive impairment and behavioral alterations [41]. Neuropsychological evaluations identified impairments in memory and executive function, highlighting the necessity for ongoing mental assistance. A thorough rehabilitation program demonstrated its efficacy in a chronic neurological Lyme disease case study, highlighting successful outcomes [42]. The patient, who continued to have symptoms while receiving antibiotic medication, showed substantial functional improvement through personalized rehabilitation programs, emphasizing the significance of a multidisciplinary approach to care [43].

RETRACTED

Managing neurological problems arising from infectious infections is changing, emphasizing precision medicine, specific medicines, and novel approaches. Progress in diagnostic tools and therapeutic techniques enhances the results for persons who are impacted [44]. Various factors influence the prognosis, and the long-term consequences may involve cognitive, behavioral, and functional impairments. Rehabilitation and supportive care are crucial in maximizing the quality of life. Thorough and continuous monitoring allows for the continuing evaluation and adjustment of treatment strategies [44]. By constantly refining our comprehension of the intricate interplay between infectious agents and the nervous system, healthcare practitioners can augment treatment techniques and boost the long-term prognosis for persons experiencing neurological symptoms of contagious disorders [45].

Challenges and future directions

The neurological symptoms resulting from viral infections present intricate difficulties in comprehending the fundamental mechanisms and executing efficient therapy measures. This section explores the present challenges in understanding and dealing with these occurrences. It suggests possible directions for future research and the development of treatments.

Elaborateness of Host-Pathogen Interactions

The complex interaction between pathogens and the neurological system poses a significant obstacle. The wide array of pathogens, including bacteria, viruses, and parasites, display diverse methods of invading and causing damage to the nervous system [41]. Understanding the intricate host-pathogen interactions at the molecular and cellular levels is essential for developing precise therapies.

Variability in Clinical Presentations

The diverse characteristics of neurological symptoms introduce intricacy to diagnosing and treating the condition. Various pathogenic microorganisms might cause comparable clinical manifestations. However, a solitary infectious agent can result in a wide range of neurological consequences [42]. Understanding the precise mechanisms behind these variances continues to be a problem, requiring an individualized approach to therapy.

RETRACTED

Delays and Uncertainties in the Diagnostic Process

Delays and uncertainty sometimes hinder the prompt and precise identification of neurological problems in the diagnostic process. The overlap of symptoms causes delays in identifying the causative agents, specialized testing requirements, and difficulties accessing suitable healthcare services [47]. This delay can impact the effectiveness of therapeutic therapies and worsen the severity of neurological consequences.

Insufficient Comprehension of the Enduring Repercussions

Understanding infectious illnesses' long-term effects on the neurological system still needs to be improved. Although specific treatments can alleviate immediate symptoms, the persistent hurdles lie in understanding and managing the long-term neurological consequences and underlying mechanisms [48]. It is crucial to clarify the elements that impact post-infectious cognitive impairment, persisting neuropathies, and chronic inflammatory states [48].

Absence of Uniform Treatment Protocols

The need for standardized treatment protocols for different infectious agents that contribute to neurological symptoms impedes the provision of appropriate patient care [49]. The need to create thorough and evidence-based treatment protocols arises from other therapeutic methods that depend on individual diseases, changes in patient populations, and changing resistance patterns [50].

Challenges in Modulating the Immune System

A careful and personalized strategy is required to handle abnormal immune responses while minimizing the risk of problems associated with immunosuppression [4]. Newly identified and previously known disease-causing microorganisms becoming more prevalent or resurfacing are emerging and re-emerging pathogens. The rise and resurgence of infectious organisms, driven by globalization, climate change, and antibiotic resistance, provide additional obstacles [51]. Newly discovered infections may have surprising tendencies to affect the nervous system and cause disease, necessitating the quick adjustment of diagnostic and treatment approaches to manage growing public health risks [52].

Disparities in Resources and the Availability of Healthcare

Inequities in healthcare resources, both on a worldwide scale and within specific locations, contribute to discrepancies in the availability of specialized care for neurological symptoms [52]. The deployment of new diagnostic technology, therapeutic interventions, and rehabilitation services may be hindered by a lack of resources, especially in locations with limited resources.

Limited Comprehension of Neuroinflammatory Mechanisms

The complex mechanisms involved in neuroinflammation during viral illnesses still need to be comprehended. Understanding the intricacies of inflammatory cascades, the function of particular cytokines, and the complex interaction between immune cells and brain tissues is crucial for developing precise anti-inflammatory approaches [53].

RETRACTED

Ethical and Social Implications

The ethical implications of researching viral diseases with neurological symptoms, particularly among disadvantaged populations, provide significant hurdles. Addressing ethical issues and ensuring fair healthcare procedures is crucial to progress in scientific knowledge and medical treatments [42].

Prospects for Future Research and Therapeutic Approaches

Utilizing multi-omics technologies, including genomes, transcriptomics, proteomics, and metabolomics, can provide a thorough comprehension of host-pathogen interactions. By integrating this data, we can uncover complex genetic patterns linked to specific neurological symptoms, which can be used to guide the development of tailored therapies [43]. Implementing personalized medicine strategies can improve the effectiveness of treatments by tailoring them to particular patients. Incorporating individualized patient characteristics, such as genetic predisposition, immunological reactions, and pathogen characteristics, will enhance the creation of tailored treatment plans optimized for various infectious diseases and neurological conditions [44]. The development of antiviral drugs that can target several virus families could significantly transform the treatment field. To overcome the difficulties posed by quickly mutating viral pathogens and emerging infectious threats, it is crucial to create agents that have a wide range of antiviral activity, can easily penetrate the CNS, and exhibit minimal resistance profiles [54]. The research is centered on refining immune regulation strategies to enhance the effectiveness of treatment interventions in illnesses characterized by immunological-mediated neurological consequences. To improve treatment strategies for disorders such as GBS and autoimmune encephalitis, it is crucial to identify precise immunomodulatory targets, determine the optimal length of therapy, and minimize potential adverse effects [34].

Neuroimaging technologies, such as fMRI, diffusion tensor imaging, and molecular imaging, have made it possible to observe and measure small changes in neural tissues. These technologies enhance our comprehension of the effects of viral illnesses on the CNS and aid in the prompt identification of neurological problems [12]. Directing neuroprotective techniques towards reducing neuronal damage is a developing field of study. Discovering medicines that can protect brain function, regulate neuroinflammation, and stimulate neuroregeneration could substantially affect the long-term prognosis of persons with viral disorders that affect the nervous system [24]. Incorporating AI and machine learning algorithms into diagnostic and therapeutic decision-making processes can improve efficiency and precision [34]. The utilization of AI in forecasting disease progressions, examining intricate datasets, and enhancing therapy algorithms has the capacity to transform clinical management. Creating cooperative international research programs that specifically target viral diseases and their neurological effects is essential [15]. International collaboration in sharing data, resources, and experience can accelerate the detection of newly developing viruses, improve diagnostic skills, and promote the creation of treatment options that can be universally used [16].

RETRACTED

Telemedicine platforms can be integrated into neurological care to tackle issues associated with resource inequities and limited access to specialized services. Telemedicine enables the provision of medical consultations, monitoring, and follow-up care from a distance, especially in areas where healthcare infrastructure is lacking [54]. It is crucial to establish strong ethical guidelines for doing research that involves infectious diseases and neurological consequences. When considering ethics, it is essential to prioritize including a wide range of populations, ensuring that permission is given with full knowledge, and addressing any potential social and cultural consequences. Implementing ethical norms will promote conscientious and fair research techniques [27]. The complex nature of neurological symptoms caused by viral diseases requires a comprehensive and collaborative treatment involving multiple disciplines. Future research should prioritize precision medicine, cutting-edge diagnostics, and revolutionary therapeutic approaches [36]. Cooperative endeavors, both on a worldwide and community scale, are crucial for tackling resource inequalities and expanding our knowledge of infectious disorders that affect the nervous system [39]. By effectively addressing these obstacles and embracing innovative research pathways, the scientific community may lay the groundwork for revolutionary progress in diagnosing and treating neurological problems linked to infectious diseases.

## Conclusions

Recent instances investigating the neurological symptoms of viral diseases have offered valuable insights into the complicated issues of comprehending and treating these ailments. The wide range of disease-causing agents and their complex interactions with the neurological system emphasize the importance of ongoing research efforts. The key findings highlight the diverse range of clinical manifestations, intricate diagnostic challenges, and the subtle nature of therapy approaches. Continuing research is crucial as we deal with the complexities of host-pathogen interactions and tackle the difficulties related to diagnosis delays, treatment uncertainty, and long-term effects. Progress in integrated multi-omics techniques, precision medicine, and neuroprotective treatments presents great opportunities for improving diagnostic accuracy and enhancing therapy results. The significance of collaborative worldwide research endeavors, ethical frameworks, and the incorporation of cutting-edge technologies cannot be emphasized enough. By promoting dedication to continuous inquiry and embracing new research avenues, we are better equipped to further our comprehension of infectious diseases that impact the nervous system and optimize patient outcomes in this rapidly evolving and demanding field.
